# Incidence and Predictive Factors of Tibial Fracture with Occult Posterior Ankle Fractures

**DOI:** 10.1155/2021/4392595

**Published:** 2021-12-08

**Authors:** Dafeng Wang, Jie Yang, Xiaomin Dong, Shengtuo Zhou, Chaonan Wang

**Affiliations:** Department of Orthopedics, Wenzhou People's Hospital, Wenzhou 325000, Zhejiang, China

## Abstract

**Background:**

Few studies exist on the predictive factors of tibial fractures with hidden posterior ankle fractures.

**Objective:**

To study the incidence and predictive factors of tibial fractures with occult posterior ankle fractures.

**Methods:**

Tibial fracture patients were prospectively selected who were admitted to our hospital from January 2016 to May 2021 and their general clinical data, X-ray images, CT images, and other imaging data were collected and then divided them into posterior malleolus fracture group and nonposterior malleolus fracture group according to the presence or absence of posterior malleolus fractures. Multivariate regression analysis and receiver operating curves (ROC) were performed to analyze the influencing factors of tibial fracture with occult posterior ankle fracture.

**Results:**

CT showed that 25 (13.44%) patients had occult posterior ankle fractures among 186 patients with tibial fracture. There was no significant difference in gender, age, and locations of tibial fracture between the two groups (*P* > 0.05). There were statistical differences in the types, locations, and lengths of patients with tibial fracture but without posterior malleolus fractures. The length of the tibia fracture group was significantly lower than the tibia with posterior ankle fracture group (*P* < 0.05). Logistics regression analysis showed that tibial fracture with occult posterior ankle fracture was not significantly correlated with gender, age, and location of tibial fracture (*P* > 0.05), but was significantly correlated with tibial fracture type, location, and length (HR = 1.830, *P*=0.035; HR = 5.161, *P*=0.004; HR = 1.126, *P*=0.030). The ROC curve showed that the AUC of length of tibial fracture with occult posterior ankle fracture was 0.599. The YD index suggested that the best cut point for the prediction of tibial fracture with occult posterior ankle fracture was above 13.18%. The sensitivity and specificity of spiral tibial fracture and distal 1/3 tibial fracture for prediction were 88.00% and 63.35%, 92.00%, and 58.39%, respectively, which was significantly higher than that of tibial fracture length (*P* < 0.05).

**Conclusion:**

Patients with tibial fractures have a higher incidence of occult posterior ankle fractures. Spiral tibial fractures and distal 1/3 tibial fractures have a higher predictive value for tibial fracture with occult posterior ankle fractures and can help clinical detection as soon as possible, which is a more accurate and appropriate treatment.

## 1. Introduction

Tibia fractures and malleolus fractures are common in clinical practice. Tibia fractures mostly presented with spiral fractures of the lower 1/3 segment, and tibial fracture is a common fracture type in clinic [1], frequently combined with occult posterior ankle fracture, which seriously affects the patient's lower limb function. During treatment, tibial fractures combined with occult posterior ankle fractures usually require posterior ankle fracture fixation on the basis of fixation of tibial fractures [2]. Tibial fractures combined with occult posterior ankle fractures are easily missed in the clinical diagnosis. Therefore, the incidence of clinical tibial fractures with occult posterior ankle fractures is much lower than the actual incidence. If missed diagnosis occurs, failure to properly treat ankle fracture components during treatment may lead to further displacement and subsequent ankle incoordination, which has been shown to affect the patient's prognosis [3–5]. Taken together, effectively mastering the epidemiological status of tibial fracture combined with occult posterior ankle fracture and effectively identifying the high-risk population of tibial fracture combined with occult posterior ankle fracture by mastering the high-risk factors of tibial fracture combined with occult posterior ankle fracture is of great significance to improve the prognosis of patients with tibial fracture combined with occult posterior ankle fracture. The present study recruited 186 patients with tibial fractures, performed ankle CT image detection, assessed the incidence of tibial fractures with occult posterior ankle fractures, and recorded the clinical data of patients to identify the predictive impact of tibial fractures with occult posterior ankle fractures.

## 2. Materials and Methods

### 2.1. General Data

Patients with tibial fractures in our hospital during January 2016 and May 2021 are retrospectively analyzed. The inclusion criteria are as follows: (1) all patients were diagnosed as tibial fractures; (2) all patients received X-ray and CT examinations; (3) all patients received CT examinations of ipsilateral ankles. Exclusion criteria: (1) lack of clinical data and no CT examination; (2) fractures that mainly involve the knee joint (tibial plateau fractures); (3) fractures that mainly involve the ankle joint (single, double, and three-toe ankle fractures); (4) fractures of patients above 65 years or unhealed fractures; (5) congenital dysplasia, neuromuscular diseases, infections, etc.; (6) bone tumors and other diseases that may change the normal anatomy of skeletal and muscle; (7) comminuted tibial shaft fractures; (8) fractures without CT images or radiographs (excluding the full length of the tibia and fibula) of the ipsilateral ankles. 186 patients were enrolled, including 135 men (72.58%) and 51 women (27.42%). This study was reviewed and approved by the Hospital Ethics Committee. The informed consents were signed by all study participants.

### 2.2. Methods

All patients received X-ray examinations after admission and were given intramedullary nail fixation according to the fracture situation. All patients received CT or MRI examinations at the ankle joint to determine if there were ankle fractures. The general clinical data and tibial fracture were recorded. All data were jointly reviewed and determined by three orthopedic surgeons.

### 2.3. Observation Indicators

The general clinical data and tibial fracture were recorded. (1) The length of tibial fractures: according to the X-ray and CT images and the proportion of the tibia length occupied by the calculator is recorded as the tibia fracture length. (2) Type of tibial fracture: according to the imaging images, the fracture is transverse, oblique, or spiral, and at least two types of fractures are recorded as complex.

### 2.4. Statistical Methods

Statistical analysis was performed using SPSS 25.0 version statistical software, measurement data was expressed by ($\bar{x}$ ± *s*), comparison between groups was by independent sample *t*-test, count data was expressed by ((*n*)%), and difference between groups was compared by *χ*^*2*^ test. Multivariable logistics regression analysis was performed to explore the influencing factors of fractured bone fracture combined with occult postcomplication fracture; we also used the receiver operator characteristic (ROC) curve to evaluate the prediction performance, calculate the area under the curve (AUC), and apply the Youden index aiming to find the best cutoff point. *P* < 0.05 means the difference is statistically significant.

## 3. Results

### 3.1. Comparison of General Information of the Two Groups of Patients

186 patients with tibial fractures were collected, including 25 patients with occult posterior ankle fractures, accounting for 13.44%. According to the presence or absence of posterior malleolus fractures, they were divided into posterior malleolus fracture group (25 cases) and posterior malleolus fracture group (161 cases). There was no statistical difference in gender, age, and tibial fracture orientation between the two groups of patients (*P* > 0.05). There were statistical differences in the types, locations, and fracture lengths of tibial fractures. The length of fractures of tibia in patients without posterior malleolus fractures was significantly lower than that of posterior malleolus fractures. The difference was statistically significant (*P* < 0.05) (see Table 1 for details).

### 3.2. Logistic Regression Analysis of Influencing Factors of Tibial Fracture with Occult Posterior Ankle Fracture

Logistics regression analysis results showed that tibial fractures with occult posterior ankle fractures were not significantly correlated with gender, age, and tibial fracture location (*P* > 0.05), but were significantly correlated with tibial fracture types, tibial fracture locations, and tibial fracture lengths (*HR* = 1.830, *P*=0.035; *HR* = 5.161, *P*=0.004; HR = 1.126, *P*=0.030) (see Tables 2 and 3 for details).

### 3.3. The ROC Curve of Tibial Fracture Length on the Prediction of Tibial Fracture Combined with Occult Posterior Ankle Fracture

The ROC curve shows that the tibial fracture length used to predict the AUC of tibial fracture combined with occult posterior malleolus fracture is 0.599; Youden index suggests that the optimal cutoff point of tibial fracture length predicted tibial fracture combined with occult posterior malleolus fracture is >13.18% (see Figure 1).

### 3.4. The Diagnostic Value of the Spiral Tibial Fracture, Distal 1/3 Tibial Fracture, and Tibial Fracture Length in Predicting the Cutoff Value of Tibial Fracture Combined with Occult Posterior Ankle Fracture

The sensitivity and specificity of spiral tibial fractures and distal 1/3 tibial fractures for the prediction of tibial fractures with occult posterior ankle fractures were 88.00% and 63.35%, 92.00%, and 58.39%, respectively, with statistical significance (*P* < 0.05) (see Table 4) (Figures 2 and 3).

### 3.5. Illustration of a Typical Case

Spiral fracture of the lower end of the left tibia, with occult posterior malleolus fracture, and transverse fracture of the right middle tibia, without occult posterior malleolus fracture, are shown in Figures 2 and 3.

## 4. Discussion

It has been revealed that posterior malleolus fractures and tibial shaft fractures often occur in clinical practice simultaneously [6, 7]. The incidence of such combined injuries is even as high as 39%–49%. It has been found that the identification of posterior ankle injuries is important for correct preoperative planning and appropriate postoperative physical therapy. During treatment of tibial fractures, neglecting posterior ankle fractures may result in iatrogenic displacement [8, 9]. Early identification of patients with tibial fractures combined with occult posterior ankle fractures can prevent posterior ankle fractures during intramedullary nailing or postoperative further displacement due to insufficient protection [10, 11]. However, during clinical diagnosis and treatment, tibial fractures and posterior ankle fractures are easily missed [12]. The first reason is that most ankle fractures are hidden fractures, and it is difficult to diagnose these fractures by X-ray; Most doctors only notice the obvious displacement of tibial shaft fractures, but usually do not take into account the possible ankle fracture, and the first X-ray film usually does not include the ankle joint, so the ankle fracture is missed. Therefore, according to the characteristics of tibial fractures, finding effective predictive factors for posterior malleolus fractures will help patients undergo more effective surgical treatment and improve their prognosis.

In this study, 25 cases (13.44%) of 186 patients with tibial fractures had occult posterior ankle fractures. The results of logistics regression analysis showed that tibial fractures with occult posterior ankle fractures were not correlated with gender, age, and tibial fracture position (*P* > 0.05), but were significantly correlated with the type of tibial fracture, the location of tibial fracture, and the length of tibial fracture (HR = 1.830, *P*=0.035; HR = 5.161, *P*=0.004; HR = 1.126, *P*=0.030). The AUC of tibial fracture length to predict tibial fracture with occult posterior ankle fracture is 0.599; Youden index suggests that the best cutoff point for tibial fracture length to predict tibial fracture with occult posterior ankle fracture is >13.18%.

When the foot is in a forward or backward rotation position, external force is applied to the talus due to rotation or valgus, which may damage the inferior tibiofibular ligament [10, 13, 14]. One side of this ligament is connected to the distal posterior edge of the tibia, the posterior malleolus. The posterior malleolus fracture is caused by avulsion of the inferior tibiofibular ligament. However, the mechanism of tibial fracture combined with posterior ankle injury is still controversial. Some studies have pointed out [15] that when tibial shaft fracture occurs, the lateral calf muscles contract, causing excessive flexion of the ankle joint plantar, and the talus compresses the posterior edge of the tibial fossa, causing ankle fracture. Studies [16] have also pointed out that the mechanism of injury is due to inertial rotation during forward movement when fixing the ankle joint, which leads to spiral fracture of the weak part involving the distal 1/3 of the tibia. The fracture line runs from the lower medial to the upper lateral. Ankle fractures are caused by shearing of the talus during movement when the foot is suddenly fixed or an avulsion fracture caused by the traction between the ankle and the posterior tibiofibular ligament. Therefore, fractures of the distal third of the tibia and spiral fractures are more likely to cause posterior malleolus fractures. The study of Tsai CE et al. [17] also pointed out that there is a significant correlation between fractures of the distal 1/3 of the tibia and spiral fractures and tibia fractures combined with posterior malleolus fractures. In order to further confirm the predictive performance of distal tibial 1/3 fractures and spiral fractures for tibial fractures combined with occult posterior malleolus fractures, the ROC curve results of distal tibial 1/3 fractures, spiral fractures, and tibial fracture lengths showed that the use of tibial spiral fractures, fractures of the distal 1/3 of the tibia, have high predictive value for tibial fractures combined with occult posterior malleolus fractures. The AUCs are 0.757 and 0.752, respectively, which are significantly higher than 0.599 of the tibial fracture length (*Z* = 1.995, *P*=0.046; *Z* = 2.048, *P*=0.041); the sensitivity of tibial spiral fracture and distal tibial 1/3 fracture to tibial fracture combined with occult posterior malleolus fracture is 88.00% and 92.00%, respectively, which is consistent with the results of Huang et al. [5].

Of course, this study also has certain limitations. We use CT as the gold standard for the diagnosis of posterior ankle fractures. Studies [2] have pointed out that, in 7 patients, after CT scan results are uncertain, 4 cases of posterior ankle fractures were confirmed by MRI. Therefore, although the observed incidence of concomitant ankle injury is higher than previous studies, the actual incidence may actually be higher if other imaging modalities (such as MRI) are used.

In summary, patients with tibial fractures have a higher incidence of occult posterior ankle fractures. Spiral tibial fractures and distal 1/3 tibial fractures have a high predictive value for tibial fractures with occult posterior ankle fractures, which can help clinically identify patients with tibial fractures and occult posterior ankle fractures as early as possible, and then take more accurate and appropriate treatment.

## Figures and Tables

**Figure 1:** The ROC curve of tibial fracture length on the prediction of tibial fracture combined with occult posterior ankle fracture.

**Figure 2:** Patients A: 56 years old, male, spiral fracture of the lower end of the left tibia, with occult posterior malleolus fracture.

**Figure 3:** Patients B: 31 years old, male, transverse fracture of right middle tibia, without occult posterior malleolus fracture.

**Table 1:** Comparison of general clinical data between the two groups ((*n*)%, ‾*χ* ± *s*).

Project		No posterior malleolus fracture group (161 cases)	Posterior malleolus fracture group (25 cases)	*χ* ^2^ */t*	*P*
Gender	Male	116 (72.05)	19 (76.00)	0.170	0.680
	Female	45 (27.95)	6 (24.00)		
Age (years)		47.53 ± 11.79	48.39 ± 10.96	−0.342	0.732
BMI (kg/m)^2^		29.57 ± 3.78	29.48 ± 3.43	0.112	0.911
Tibia fracture location	Left side	84 (52.17)	12 (48.00)	4.364	0.179
	Right	77 (47.83)	12 (48.00)		
	Bilateral	0 (0.00)	1 (4.00)		
Types of tibial fractures	Horizontal	60 (37.27)	0 (0.00)	64.876	<0.001
	Tilt	56 (34.78)	3 (12.00)		
	Spiral	23 (14.29)	22 (88.00)		
	Complex	22 (13.66)	0 (0.00)		
Tibia fracture location	Near 1/3	43 (26.71)	1 (4.00)	22.564	<0.001
	Central 1/3	52 (32.30)	1 (4.00)		
	Distal 1/3	66 (40.99)	23 (92.00)		
Tibia fracture length (%)		13.19 ± 4.81	15.24 ± 4.67	−2.087	0.038

**Table 2:** Logistics regression analysis assignment table.

	Factors	Assignment description
X1	Gender	Male = 1, female = 0
X2	Age	Continuous variable
X3	Position of tibial fracture	Left = 1, right = 2, bilateral = 3
X4	Type of tibial fracture	Lateral = 1, tilt = 2, spiral = 3, complex = 4
X5	Fracture position of tibia	Proximal 1/3 = 1, middle 1/3 = 2, distal 1/3 = 3
X6	Fracture length of tibia	Continuous variable
Y	Occult posterior malleolus fracture	Yes = 1, no = 0

**Table 3:** Logistic regression analysis results of influencing factors of tibial fractures with occult posterior ankle fractures.

Factors	*β*	S. E.	Wald	*P*	HR	95 CI	
						Lower limit	Upper limit
Gender	0.444	0.580	0.586	0.444	1.559	0.500	4.861
Age	0.001	0.023	0.001	0.977	1.001	0.957	1.046
Position of tibial fracture	0.451	0.463	0.948	0.330	1.570	0.633	3.891
Type of tibial fracture	0.589	0.280	4.425	0.035	1.803	1.041	3.123
Fracture position of tibia	1.641	0.569	8.324	0.004	5.161	1.693	15.737
Fracture length of tibia	0.119	0.055	4.726	0.030	1.126	1.012	1.253

**Table 4:** Diagnosis value of spiral tibial fracture, distal 1/3 tibial fracture, and tibial fracture length for the prediction of cutoff value of tibial fracture combined with occult posterior ankle.

Detection methods	Accuracy	Sensitivity	Specificity	Positive predictive value (%)	Negative predictive value (%)
Helical tibial fracture	66.67%^a^	88.00%^a^	63.35%^a^	27.16	97.14^a^
1/3 fracture of distal tibia	62.90%^a^	92.00%^a^	58.39%	25.56	97.92^a^
Fracture length of tibia	51.08%	64.00%	49.07%	16.33	89.77

*Note.* Compared with the fracture length of tibia, *P* < 0.05.

## Data Availability

The simulation experiment data used to support the findings of this study are available from the corresponding author upon request.
